The article "Biogenic Analysis of the Effect of TERC on Cell Proliferation and Migration of Oral Squamous Cell Carcinoma under Digital Minimally Invasive Treatment" was retracted in 2023. Reasons: unreliable results or conclusions; lack of ethics approval or compliance; concerns about the data; concerns about the peer review.

# Biogenic Analysis of the Effect of TERC on Cell Proliferation and Migration of Oral Squamous Cell Carcinoma under Digital Minimally Invasive Treatment

**DOI:** 10.1155/2022/2102795

**Published:** 2022-08-18

**Authors:** Wenao Chen, Zilong Zhang, Yiyao Jin, Ruijie Zeng, Xi Sun, Zihan Zhou, Kabna Kasim, Joshua Grant, Vumika Kuraki, Felix Schmid, Gabin Lucas

**Affiliations:** ^1^I.M. Borovsky Institute of Dentistry, I.M. Sechenov First Moscow State Medical University, Moscow 119991, Russia; ^2^Stomatological Hospital of Anhui Province, Anhui Medical University, Hefei, Anhui 230031, China; ^3^University of Kragujevac, Kragujevac, Serbia; ^4^University of Melbourne, Melbourne, Australia; ^5^Kobe University, Kobe, Japan; ^6^Carleton University, Ottawa, Canada; ^7^University of British Columbia, Vancouver, Canada

## Abstract

**Objective:**

To investigate the correlation between TERC gene and cell proliferation and migration of oral squamous cell carcinoma.

**Methods:**

By comparing the traditional surgical treatment with the minimally invasive treatment of digital technology, the influence of Shengxin analysis method on the proliferation and migration of oral squamous cell carcinoma cells was analyzed.

**Results:**

Digital technology minimally invasive treatment has a great impact on the operation and survival rate of patients. TERC has a significant impact on the proliferation and migration of oral squamous cell carcinoma cells. Digital technology minimally invasive treatment can prevent TERC from great changes.

**Conclusion:**

TERC under the minimally invasive treatment of digital technology has little effect on the proliferation and migration of oral squamous cell carcinoma cells. It can promote the proliferation of oral squamous cell carcinoma cells. The inhibitors of migration and invasion can play an effective role in antiproliferation.

## 1. Introduction

With the improvement of living standards, people's quality of life has also changed. People are also increasingly concerned about health. They will have regular physical examination every year to pay attention to any problems that may occur in their physical functions. However, there are many diseases that cannot be found in the early stage. It is possible that the occurrence of a disease will cause problems in other organs. Today, many cancers cannot be cured. People are suffering from cancer, both physically and at home. With the change of living conditions, people are also pursuing some so-called “game,” in which many bacteria and viruses are eaten into the stomach. What cannot be absorbed by itself will lead to physical problems, such as oral squamous cell carcinoma, which refers to the malignant tumor occurring in the mouth and mainly composed of squamous cells. It is the most malignant and harmful tumor in the head and neck, accounting for 50% of the cases of head and neck squamous cell carcinoma. How does the mode of medical care integration affect oral squamous cell carcinoma? Jia (2022) and others analyzed the impact of integrated management intervention on oral squamous cell carcinoma patients and discussed their oral health, quality of life, and psychological status. The results showed that it could effectively improve their quality of life and psychological enthusiasm and more effectively alleviate patients' anxiety [1]. We can more accurately understand how to treat the proliferation and migration of cancer cells. Feng (2022) and others analyzed and mechanism it and studied the inhibitory effect of interleukin on the proliferation of cancer cells [2]. In order to better control and inhibit the dispersion of cancer cells, Yingying (2022) and others used long-chain noncoding RNA col11a1-208 to analyze the effect of its cell proliferation and invasion. Col11a1-208 can promote its cell proliferation and invasion ability and play an important role in the occurrence and progress [3]. The progress of medicine and the development of scientific research, compared with the previous incurable diseases, are many. First, now, we are also studying how to treat them to alleviate the pain of patients faster, but there are also many diseases that deteriorate, which are closely related to psychological effects. The strength of psychological quality is crucial to physical function. Li (2022) and others analyzed and discussed the impact of their postoperative psychological state and used dialectical behavior therapy to effectively promote the positive growth of their postoperative patients' traumatic psychology, improve their psychological state, and improve their survival level [4].

The article "Biogenic Analysis of the Effect of TERC on Cell Proliferation and Migration of Oral Squamous Cell Carcinoma under Digital Minimally Invasive Treatment" was retracted in 2023. Reasons: unreliable results or conclusions; lack of ethics approval or compliance; concerns about the data; concerns about the peer review.

There are about 100000 new oral cancer patients in the world every year. A large number of patients with oral cancer are mainly of high malignancy. The treatment is mainly a combination of surgery, radiotherapy, and chemotherapy. However, the survival rate of patients within 5 years fell to 50%. In this regard, Lin (2022) and others analyzed the value-added of their disease, and the results showed that this research and analysis could inhibit the value-added of cancer cells and promote cell apoptosis [5]. For the change of postoperative nutritional status of patients and the analysis of its influencing factors, Mair Haba (2022) and others analyzed the status and influencing factors during the treatment process, so as to better understand the situation of postoperative patients [6]. In the process of clinical treatment, the clinical characteristics of oral squamous cell carcinoma cells are variable. For this, Zhao (2022) and others discussed the correlation between their characteristics and prognosis, which can make the difference between the treatment of their disease and prognosis clearer [7]. In order to understand the important role of early epithelial stromal transformation in regulating the dryness and metastasis of cancer cells, Zhu (2022) and others analyzed the role and mechanism of its transformation, which can play a key role in the treatment of patients [8]. In this study, in order to better treat and control the proliferation and migration of oral squamous cell carcinoma cells, TERC under the minimally invasive treatment of digital technology was used to conduct genetic analysis and research.

## 2. Patient Information

### 2.1. General Information

80 patients with oral squamous cell carcinoma treated in our hospital from 2018 to 2022 were selected, including 58 males and 22 females. The age of male patients is 32~68 years old, and the age of female patients is 37~66 years old. Among them, 18 cases were tongue lesions, 22 cases were palate lesions, 11 cases were buccal lesions, 7 cases were floor of mouth lesions, and 22 cases were lesions in other parts.

### 2.2. Inclusion and Exclusion Criteria

1. All patients were patients with simple oral squamous cell carcinoma, including oral squamous cell carcinoma caused by different reasons such as heredity, environment, and living habits
2. All other organs of all patients have complete structures and are normal after medical examination
3. All physical indicators of all patients were normal
4. Those who did not return to the hospital on time were excluded in the observation stage
5. Patients who did not comply with medication were excluded in the observation stage
6. All patients have no infectious diseases or are allergic to drugs for the treatment of the disease

## 3. Method

### 3.1. Routine Surgical Treatment

Oral squamous cell carcinoma is mainly treated by surgery for a wide range of excised lesions. Because of oral squamous cell carcinoma, the main purpose of surgery is functional repair. For example, if squamous lesions occur in tongue or buccal mucosa, they can be directly closed and sutured if they are removed early. For extensive invasion, there must be good repair methods, such as taking the forearm flap or taking the lateral oral flap. When the squamous cell carcinoma develops seriously, it may be necessary to cut off part of the jaw, including the maxilla, mandible, and oropharynx, which will cause the loss of oral function. In this case, more complex repair methods will be used to restore the patient's oral function while removing the lesion.

The article "Biogenic Analysis of the Effect of TERC on Cell Proliferation and Migration of Oral Squamous Cell Carcinoma under Digital Minimally Invasive Treatment" was retracted in 2023. Reasons: unreliable results or conclusions; lack of ethics approval or compliance; concerns about the data; concerns about the peer review.

### 3.2. Digital Technology Minimally Invasive Treatment

Use digital technology to analyze the precise focus before operation, scan and image the maxillofacial bone, and make a personalized operation plan according to the results. Using minimally invasive surgery, according to the preoperative plan, the squamous cell carcinoma cells in the oral cavity were accurately removed and neck lymph node dissection, and then microsurgical vascular anastomosis and defect repair were performed. In the early stage, there can be no symptoms. With the progression of the tumor, local masses can appear, accompanied by ulceration and easy bleeding. Surgical treatment should be the first choice after the diagnosis of oral cancer. The specific surgical method also needs to be determined according to the size of the tumor, the scope of invasion, and whether there is metastasis in other parts. If there is no metastasis and the focus is small, it can be minimally invasive without sweeping other tissues.

### 3.3. Shengxin Analysis

Bioinformatics analysis refers to the analysis of biological information, which reflects the state and mode of biological movement. Biological information is mainly biological genetic genes. All kinds of tumors and cancers are diseases that cause cells to stimulate the formation of new organisms due to DNA mutations. With the development of gene sequencing technology, the impact of TERC gene on the proliferation and migration of oral squamous cell carcinoma cells was identified through biological information analysis. The bioscience analysis process is shown in Figure 1.

Analyze the data of its cancer patients, input the data into the big data platform, filter and sort out the gene expression data through the big data platform to obtain the available data, screen the TERC gene of its cell cancer, analyze and discuss the impact of TERC on the proliferation and migration of cancer cells after minimally invasive treatment with digital technology, and finally draw a conclusion. This method is not only the fastest but also the most effective treatment method. It can more intuitively carry out a more specific biochemical analysis of oral squamous cell carcinoma cells and have a deeper understanding of the patient's condition, so that the treatment is more conducive to the patient's treatment plan.

### 3.4. Statistical Methods

The study set up the conventional surgical treatment group and the digital technology minimally invasive treatment group, the statistical data are different according to the different treatment of patients. According to the statistical information obtained in the above treatment methods, group analysis was carried out to analyze the statistical correlation and corresponding relationship between the data. The statistical software platform is IBM SPSS 24.0 data analysis platform, and the bivariate *t*-test method is used to compare the differences of data. When *t* < 10.000, it is considered that there is statistical difference in the data and the significance *p* value of the statistical data. When *p* < 0.05, it is considered that the statistical results are credible, and when *p* < 0.01, it is considered that the statistical results have significant statistical significance.

The article "Biogenic Analysis of the Effect of TERC on Cell Proliferation and Migration of Oral Squamous Cell Carcinoma under Digital Minimally Invasive Treatment" was retracted in 2023. Reasons: unreliable results or conclusions; lack of ethics approval or compliance; concerns about the data; concerns about the peer review.

## 4. Results

### 4.1. Comparison of Patients' Surgical Impact under Different Methods

Oral mucosal epithelium belongs to squamous epithelium. The cancer that occurs in oral mucosal epithelium is called oral squamous cell carcinoma, namely, oral squamous cell carcinoma. Oral squamous cell carcinoma is a common and harmful malignant tumor in the mouth. Now, patients with oral squamous cell carcinoma are treated in groups, and the effects of the two methods on surgical focus location, intraoperative focus clearance, and postoperative recurrence rate are compared. The data are made into Table 1 as follows.

As shown in Table 1, the location of the focus of patients using digital technology minimally invasive treatment is more accurate than that of conventional surgery, and both the clearance rate and recurrence rate of the focus are better than those of patients undergoing conventional surgery. Make the data in Table 1 into a visual diagram, as shown in Figure 2.

In Figure 2, the digital technology minimally invasive treatment method performs well in all aspects of treatment. Compared with traditional treatment methods, digital technology minimally invasive treatment method is more effective, which is more conducive to patients to alleviate pain, improve treatment rate, and lay the foundation for survival rate. It can be considered that different treatment methods have a certain impact on the focus location, focus clearance, and recurrence rate of oral squamous cell carcinoma. The treatment method under the minimally invasive digital technology has a better effect on the treatment and prognosis of oral squamous cell carcinoma.

### 4.2. Correlation Analysis of the Effects of TERC on Cell Proliferation and Migration of Oral Squamous Cell Carcinoma under the Two Methods

In normal human cells, telomerase activity is closely regulated. Only in cells that constantly divide and clone can telomerase activity be detected. In this tumor cell, TERC gene expression increased, which indicates that TERC gene plays an important role in this cancer cell. The effects of TERC on cell proliferation and migration under the two methods are analyzed, and Table 2 and Figure 3 are obtained.

The article "Biogenic Analysis of the Effect of TERC on Cell Proliferation and Migration of Oral Squamous Cell Carcinoma under Digital Minimally Invasive Treatment" was retracted in 2023. Reasons: unreliable results or conclusions; lack of ethics approval or compliance; concerns about the data; concerns about the peer review.

It can be seen in Table 2 and Figure 3 that the value-added rate of oral squamous cell carcinoma cells using conventional surgical methods is 20% and the cell migration rate is 17.5%, while the value-added rate and migration rate of oral squamous cell carcinoma cells under the minimally invasive treatment method of digital technology are 7.5% and 5%, respectively, which is significantly lower than that of conventional surgical methods. Oral squamous cell carcinoma has many high-risk factors and complex pathogenic factors, which is conducive to the diagnosis, treatment, and prevention of oral squamous cell carcinoma, and has important clinical value.

### 4.3. Comparison of Patient Survival Rate under Different Methods

At present, the prevalence of cancer is increasing year by year, but there are also many cancers that cannot be cured. Once found, some cancers may be in the late stage of cancer, or even in the middle stage, and the survival rate is low. In this regard, the survival rate of oral cancer must be found earlier and treated in time. It also has a certain relationship with the standardization of treatment. For example, if standardized surgery is carried out and other treatments are followed up, its cure rate can be greatly improved. If it is found late or does not get standardized treatment, and the best treatment time and treatment period are delayed, its survival rate will be reduced by half. In this regard, two different treatment methods were used to compare the survival rates of the same number of patients. The survival rates of 1, 3, and 5 years were compared.  Table 3 was drawn according to the data values obtained from the analysis.

In Table 3, the number of patients with the two treatment methods is the same. According to the survival rate in different time periods, the survival rate in routine surgical treatment is also increasing year by year, and the five-year survival rate data value is about 60%. Compared with the minimally invasive treatment of digital technology, the 5-year survival rate is increased to more than 70%, which can effectively improve the survival rate and reduce mortality. According to the statistical method, there was *t* < 10.000 and *p* < 0.05 between the two comparisons of the data, which was statistically significant. In order to observe the data values in the two different treatment methods more intuitively, Figure 4 is drawn according to the data in Table 3.

As shown in Figure 4, taking one year as an example, the survival rate of traditional treatment is 80%, while the data of digital technology treatment is 93%, which has a more significant effect. In this regard, in the new information age, the application of scientific research technology in medicine is the gospel of the majority of patients, which not only improves the survival rate but also reduces the treatment time for doctors in the treatment process, provides the basis for patients in the later treatment, and reduces patients' pain. What is more, it reduces the doctor-patient disputes in the hospital, provides the basis for building a harmonious hospital environment, and greatly alleviates the contradictions between medical staff and patients.

The article "Biogenic Analysis of the Effect of TERC on Cell Proliferation and Migration of Oral Squamous Cell Carcinoma under Digital Minimally Invasive Treatment" was retracted in 2023. Reasons: unreliable results or conclusions; lack of ethics approval or compliance; concerns about the data; concerns about the peer review.

## 5. Discussion

With the acceleration of the pace of life and the increase of social pressure, more and more people suffer from cancer, and the symptoms are becoming more and more complex. In this regard, Cong (2022) and others talked about the possible mechanism of aspirin inhibiting the proliferation of its cells by inducing apoptosis [9]. At present, some drugs can inhibit the proliferation of cancer cells. All trans-retinoic acid combined with apatinib has a qualitative inhibitory effect on the proliferation of oral squamous cell carcinoma cells. Therefore, Pan et al. (2022) studied it and showed that all trans-retinoic acid combined with apatinib can inhibit the proliferation of oral squamous cell carcinoma cells by promoting cell aging and affecting cell dryness [10]. This can alleviate the suffering caused by the pain, but this relief is also to a certain extent, and cannot completely control the disease. All diseases must be treated with drugs or drugs, but the overdose of some drugs will lead to the reduction of drug resistance, which cannot achieve the desired effect. For this, Sun (2022) and others studied and analyzed the drug resistance of oral squamous cell carcinoma, activated and inhibited the proliferation of cisplatin resistant cells in oral squamous cell carcinoma, promoted apoptosis, and reduced the resistance of oral squamous cell carcinoma cells to cisplatin [11]. Yun et al. (2022) also analyzed the influence on the invasion and migration ability of its cancer cells, and vines can significantly inhibit the invasion, migration, and tumor growth ability of oral squamous cell carcinoma cells [12]. Honor et al. (2022) studied the cell cycle arrest and apoptosis of oral squamous cell carcinoma. Transfection of si-neat1 can inhibit the proliferation of oral squamous cell carcinoma cells, induce apoptosis, and cause cycle arrest [13]. Although drug treatment can alleviate this disease, it cannot be better treated in routine treatment. In the continuous updating and reform of scientific research technology, digital technology minimally invasive treatment has a certain impact on its disease, which can better treat the value-added and migration of this disease. It can better control the incidence of oral squamous cell carcinoma, slightly alleviate the pain caused by the disease, help to get a specific understanding of the development of oral squamous cell carcinoma disease, and better formulate a treatment plan in the treatment process.

The article "Biogenic Analysis of the Effect of TERC on Cell Proliferation and Migration of Oral Squamous Cell Carcinoma under Digital Minimally Invasive Treatment" was retracted in 2023. Reasons: unreliable results or conclusions; lack of ethics approval or compliance; concerns about the data; concerns about the peer review.

## 6. Summary

Based on TERC under digital technology minimally invasive treatment, this study studied the influence of cell proliferation and migration of oral squamous cell carcinoma. Through the comparison of surgical effects and survival rates of patients under different treatment methods, the influence of TERC gene changes on cell proliferation and migration was studied and analyzed. Under the new technology research, the application of digital technology minimally invasive treatment can effectively control and treat its disease. With the rapid development of precision medicine and information technology, digital technology is gradually applied to various fields of medicine, which can promote the development of medicine towards precision and minimally invasive. Improve the accuracy of diagnosis, treatment, and nursing in the treatment process, improve the effect of treatment, and reduce labor intensity. In the digital information age, medicine needs to follow rules and regulations, but also needs innovation and development to obtain more extensive applications. No matter in any field or industry, the impact of digitalization has an inseparable relationship with the development of all walks of life, which is more conducive to the progress of social economy and the rapid development of society.

## Figures and Tables

**Figure 1:** Flowchart of bioinformatics analysis of the effect of TERC gene on oral squamous cell carcinoma cells.

**Figure 2:** Comparison of surgical impact of patients under different methods.

**Figure 3:** Effect of TERC on cell proliferation and migration of oral squamous cell carcinoma under two methods.

**Figure 4:** Visualization of survival rate of patients with different treatment methods.

**Table 1:** Comparison of surgical impact of patients under different methods.

Grouping	*n*	Focus localization	Focal debridement	Recurrence rate
Routine surgical treatment	40	78%	73%	14%
Digital technology minimally invasive treatment	40	92%	95%	5%
*t*		8.523	7.675	7.936
*p*		0.015	0.012	0.023

**Table 2:** Analysis of the effect of TERC on cell proliferation and migration of oral squamous cell carcinoma under the two methods.

Grouping	*n*	Gene amplification rate	Gene migration rate
Routine surgical treatment	40	20%	17.5%
Digital technology minimally invasive treatment	40	7.5%	5%

The article "Biogenic Analysis of the Effect of TERC on Cell Proliferation and Migration of Oral Squamous Cell Carcinoma under Digital Minimally Invasive Treatment" was retracted in 2023. Reasons: unreliable results or conclusions; lack of ethics approval or compliance; concerns about the data; concerns about the peer review.

**Table 3:** Comparison of survival rate of patients with different treatment methods.

Grouping	*n*	1-year survival rate	3-year survival rate	5-year survival rate
Routine surgical treatment	40	80%	73%	61%
Digital technology minimally invasive treatment	40	93%	81%	74%
*t*		8.125	9.012	8.756
*p*		0.048	0.041	0.032

## Data Availability

The data underlying the results presented in the study are available within the manuscript.

## References

[1] Lina J., Zheng W., Yufan W., Miaoli C. (2022). Effect of integrated medical care and whole process management on patients with oral squamous cell carcinoma. *Nursing Practice and Research*.

[2] Xuemei F., Xin F., Yajie W. (2022). The role and mechanism of IL-24 in regulating the proliferation of oral squamous cell carcinoma cells through jak2/stat3 pathway. *Journal of Clinical Stomatology*.

[3] Yingying J., Xi C., Yu S., Jicheng Y., Wang X., Gang D. (2022). Effect of long-chain non coding RNA col11a1-208 on proliferation and invasion of oral squamous cell carcinoma cells. *PLA Medical Journal*.

[4] Li Zhuo W., Hong L. M. (2022). Effect of syndrome differentiation behavior therapy on post-traumatic growth and psychological state of patients with oral squamous cell carcinoma after surgery. *Journal of Northern Sichuan Medical College*.

[5] Fangliang L., Jie Z., Lixia Z., Zhengtao Y., Dong W. (2022). lncrna foxd2-as1 targeting mir-1299 inhibits proliferation and induces apoptosis of oral squamous cell carcinoma cells in vitro. *Hebei Medicine*.

[6] Maihemuti M. H., Jie B., Imiti R. S., Zhitao Y. (2022). Analysis of nutritional status changes and influencing factors in 50 patients with oral squamous cell carcinoma during treatment. *Shanghai Stomatology*.

[7] Cong Z., Yuzhi W., Min H., Yan L., Sen Y. (2022). Correlation between nkd2 gene methylation and clinical characteristics and prognosis of oral squamous cell carcinoma. *Journal of Practical Cancer*.

[8] Qingqing Z., Chen S., Jianli S., Zhenjie G. (2022). Effect and mechanism of low expression of ENPP1 on epithelial mesenchymal transformation of oral squamous cell carcinoma cells. *Chinese General Medicine*.

[9] Beibei C., Xu Y., Gao M., Yu X., Wang W., Fang W. (2022). Effect and mechanism of aspirin on proliferation and apoptosis of oral squamous cell carcinoma cells. *Journal of Qingdao University (Medical Edition)*.

[10] Xinhua P., Zhe L., Lulu Y., Guopei Z. (2022). Inhibition of oral squamous cell carcinoma cell proliferation by all trans retinoic acid combined with apatinib in vitro. *Oral Biomedicine*.

[11] Yanyan S., Tao W., Lin H., Hailian J. (2022). Effect and mechanism of lncrna ac093818.1 on cisplatin resistance of oral squamous cell carcinoma cells. *Journal of Practical Stomatology*.

The article "Biogenic Analysis of the Effect of TERC on Cell Proliferation and Migration of Oral Squamous Cell Carcinoma under Digital Minimally Invasive Treatment" was retracted in 2023. Reasons: unreliable results or conclusions; lack of ethics approval or compliance; concerns about the data; concerns about the peer review.

[12] Lei Y., Tuqiang H., Hao Z., Li H. (2022). Effect of sinomenine on invasion and migration of oral squamous cell carcinoma cells. *Journal of Clinical Stomatology*.

[13] Honor H. Z., Na Z. (2022). Effects of lncrna neat1 on cell cycle arrest, apoptosis and hippo/yap signaling pathway in oral squamous cell carcinoma cells. *Journal of Practical Stomatology*.

